The article "Changes of Intestinal Microflora in Colorectal Cancer Patients after Surgical Resection and Chemotherapy" was retracted in 2023. Reasons: signs of a paper mill; suspected computer-generated content; unreliable results or conclusions; concerns about the data.

# Changes of Intestinal Microflora in Colorectal Cancer Patients after Surgical Resection and Chemotherapy

**DOI:** 10.1155/2022/1940846

**Published:** 2022-02-24

**Authors:** Rui Huang, Ke He, Xiaopeng Duan, Jinfeng Xiao, Hanning Wang, Guoan Xiang

**Affiliations:** Guangdong Second Provincial General Hospital, Guangzhou, Guangdong 510317, China

## Abstract

**Objective:**

The change of bacterial flora structure in colorectal cancer (CRC) patients after treatment is not clear. The aim of this study was to explore the change and function of intestinal microflora in CRC before and after treatment.

**Method:**

The 16S conserved region V3+V4 of intestinal flora obtained from CRC patients was sequenced and analyzed. Alpha and beta diversity indices were used to analyze the abundance and structure of gut flora. FAPROTAX, BugBase, and Tax4Fun software were used to analyze the species phenotypes and Kyoto Encyclopedia of Genes and Genomes Ontology (KO) function pathways.

**Results:**

Total abundance and structure of species in CRC patients were significantly increased compared with healthy people (control group) (*P* < 0.05), but there was no significant difference between CRC patients before and after treatment (*P* > 0.05). There was significant difference in relative abundance of bacteria at different levels (phylum, class, order, family, genus, and species) between the CRC group with after operation (CRC_O group) and chemotherapy (CRC_C group) treatment, particularly *Prevotellaceae_UCG-001*, *Akkermansia*, *Fusicatenibacter*, *Tyzzerella_4*, *Megamonas*, etc. in genus level. The KO function analysis showed that most of the bacteria with differences were mainly involved in the biosynthesis of lipopolysaccharide (*Megamonas*, *Megasphaera*, and *Ruminococcus torques_group*), protein digestion and absorption, renin-angiotensin system pathway (*Akkermansia*, *Eubacterium_ruminantium_group*, and *Eubacterium_nodatum_group* genus), adipocytokine signaling pathway and peroxisome pathway (*Tyzzerella_4*, *Phascolarctobacterium*, *Ruminococcus_gnavus_group*), and so on.

**Conclusion:**

The abundance of intestinal microflora in CRC patients was increased significantly contrasted to healthy people, and surgery and chemotherapy were hard to reduce this phenomenon. *Megamonas* was involved in lipopolysaccharide biosynthesis and carcinogenesis in colorectal cancer. Surgery and drug treatment did not reduced lipopolysaccharide biosynthesis but increased the number of probiotic *Akkermansia* population and reduced the pathogenic bacteria *Tyzzerella_4*, participate in adipocytokine signaling pathway, and affect metabolism.

## 1. Introduction

The incidence of colorectal cancer (CRC) ranks third in the total number of cancer patients in the world, and the mortality rate ranks fourth in the global cancer-related deaths [1]. In China, 376000 new cases and 191000 deaths of CRC occur in 2015 [2], which is the fourth largest tumor in China. With the continuous improvement of living standards, and the intake of high-fat and high sugar foods, the incidence rate of CRC is increasing year by year. The onset age of CRC is gradually younger, and there are no obvious clinical symptoms in the early stage. Advanced CRC metastasizes to distal organs, leading to important organ failure and death, which seriously threatens human health [3]. Currently, the treatment strategies of CRC include surgical resection, radiotherapy, chemotherapy, targeted therapy, and emerging immunotherapy. The effective rate of surgery combined with radiotherapy and chemotherapy is as high as 70% to 80%, and the 3-year overall survival is up to 53%. With the development of tumor, the survival rate of CRC patients is also declining [4]. In addition, 20%-30% of CRC patients receiving treatment are at risk of recurrence [5]. To evaluate the risk of formation and recurrence of colorectal cancer and to seek effective treatment strategies for intestinal cancer are the focus of clinical research.

The article "Changes of Intestinal Microflora in Colorectal Cancer Patients after Surgical Resection and Chemotherapy" was retracted in 2023. Reasons: signs of a paper mill; suspected computer-generated content; unreliable results or conclusions; concerns about the data.

In recent years, many studies have shown that intestinal flora disorder is an important factor leading to CRC in addition to genetics, environment, and diet. In fact, a large number of studies have confirmed the significant changes of intestinal flora composition between CRC patients with normal one. Several bacterial species have proinflammatory and carcinogenic characteristics and are involved in the occurrence of colorectal cancer [6]. Normally, the intestinal tract of human body is rich in four bacterial groups including Hirsutella, Bacteroides, Proteus, and Actinomycetes, which regulate the body's normal nutrient absorption, metabolism, and immunity. In CRC patients, *Gram-negative* bacteria are enriched, while *Gram-positive* bacteria and *Actinomycetes* are decreased. For example, a large number of pathogenic bacteria such as *Porphyromonas*, *Colibacilli*, *Staphylococcus*, *Ackermann*, and *Methanogens* genus are detected in the intestinal tract of CRC patients, while *Bifidobacterium*, *Lactobacillus*, *Ruminococcus*, *Bacillus*, *Roseburia*, and *Treponema* genus are poor. Some scholars found that the species abundance of *Clostridium* and *Fusobacterium* is negatively correlated with tumor count. Animal model experiments show that beneficial bacteria such as high level of *Clostridium* implanted into the intestinal tract effectively reduce the burden of CRC [1, 7, 8].

The article "Changes of Intestinal Microflora in Colorectal Cancer Patients after Surgical Resection and Chemotherapy" was retracted in 2023. Reasons: signs of a paper mill; suspected computer-generated content; unreliable results or conclusions; concerns about the data.

With the development of molecular technology and the improvement of microbial genomics, the causal relationship between cancer and intestinal flora has been continuously recognized. Intestinal flora has become a key component not only in tumorigenesis but also in disease-free survival after surgery. Some scholars believe that it has a potential role in reducing postoperative inflammation and recurrence rate of CRC [9, 10]. However, there are few studies on the effect of intestinal flora on recurrence and prognosis of CRC. This study focuses on the combination of microbial sequencing and bioinformatics analysis technology to explore the changes of intestinal flora in patients with CRC before and after treatment and to analyze the impact and significance of this difference on recovery or recurrence after treatment.

## 2. Methods

### 2.1. Diagnosis and Treatment of Colorectal Cancer Patients

Patients diagnosed with CRC by digital anal examination assisted by rectal endoscopy [11] were included in the study. Some intestinal hyperplasia tissues were taken with biopsy forceps for pathological examination (including hematoxylin and eosin staining) to determine the deterioration of intestinal hyperplasia. CRC patients underwent surgical resection of tumor tissue and received chemical therapy (treated with tegafur, calcium folinate, and oxaliplatin for 5 days) one month later. Patients had no obvious discomfort during chemotherapy.

### 2.2. Collection and Treatment of Samples

From May 2019 to October 2019, a total of 17 fecal microbiological samples were collected from healthy people and patients with colon and rectal cancer, including 5 normal samples (control group). Among the intestinal microbiological samples of colorectal cancer (CRC group), there were 3 colon cancer (CC) samples and 2 rectal cancer (RC) samples. There were 3 cases of CRC samples after operation (CRC_O) and 4 cases of CRC samples after chemotherapy (CRC_C). The samples were collected with sterile fecal collection kit and sent to the sterile operation platform. Microbial DNA was extracted immediately with fecal DNA extraction kit and then stored at -20/-80°C. The extracted total DNA samples were transported to the laboratory with dry ice for subsequent amplification, library construction, and sequencing (Figure 1).

### 2.3. Sequencing and Data Processing of 16S rDNA of Intestinal Flora

The V3+V4 region of 16S rDNA was amplified by specific primers with barcode. The upstream primer was 5′-CCTACGGGNGGCWGCAG-3′ (341), and the downstream primer was 5′-GGACTACHVGGGTATCTAAT-3′ (806). The size of the amplified product was about 466 bp. QuantiFluor™ fluorometer (Promega, Madison, WI, USA) was used to quantify the DNA of samples. The purified amplified products were mixed in the same amount, connected to the sequencing connector, and the sequencing library was constructed. Illumina PE250 (San Diego, CA, USA) was used for sequencing. The raw reads obtained by sequencing were first removed by FASTP software [12], and then tags were spliced into raw reads with Fast Length Adjustment of Short Reads (FLASH) software [13]. UCHIME algorithm [14] of USEARCH software (http://www.drive5.com/) was used to filter chimera and other nonbiological data, so as to enhance the statistical reliability and biological validity of the data.

The article "Changes of Intestinal Microflora in Colorectal Cancer Patients after Surgical Resection and Chemotherapy" was retracted in 2023. Reasons: signs of a paper mill; suspected computer-generated content; unreliable results or conclusions; concerns about the data.

### 2.4. OTU Clustering and Bacterial Species Annotation

The effective reads were clustered according to sequence similarity, and the tag sequences with 100% similarity were classified as an operational tax unit (OTU). The absolute and relative abundances of each OTU in each group were calculated. The common and unique OTUs of each group were analyzed and compared. The OTU sequences were compared by SILVA software (https://www.arb-silva.de/) [15], and the bacterial population was annotated according to 97% sequence similarity.

### 2.5. Alpha Diversity Analysis

The Observed_OTUs (Sobs, species richness), Chao1 (bacterial diversity), and Abundance-based Coverage Estimator (ACE, bacterial abundance) indexes were calculated. Simpson and Shannon comprehensively reflected the species richness and evenness.

### 2.6. Beta Diversity Analysis

The Jaccard distance index was mainly based on the presence or absence of species to evaluate the difference of flora structure. Bray_curtis was based on the presence or absence of species and species abundance. Unweighted_unifrac was based on the evolutionary distance of species. Weighted_unifrac was based on evolutionary distance and species abundance. Unweighted pair group method with arithmetic mean (UPGMA) cluster tree and principal coordinate analysis (PCoA) analysis were conducted based on the above four distance indexes to observe the difference degree of microbial community structure among samples. The ANOSIM test model was used to determine the significance of the differences in the microbial community structure between groups.

### 2.7. Analysis of Intestinal Marker Bacteria in Patients with Colorectal Cancer before and after Treatment

Based on the abundance and frequency of genus in the samples, the indicator value (IndVal) of each group was calculated. The higher the value was, the more likely the genus was to be a biomarker of a group. Using “labdsv” toolkit (https://rdrr.io/cran/labdsv/) of R software, IndVal was calculated, and cross-validation was used for statistical test to screen the marker flora with *P* value less than or equal to 0.05. Linear discriminant analysis (LDA) effect size (LEFSE) was used to assist in assessing the relative abundance of bacterial taxa, and the nonparametric Kruskal-Wallis rank sum test was used to compare the significantly abundant bacterial taxa in different groups. Taxa with LDA greater than 2 and *P* value ≤ 0.05 were considered significant.

The article "Changes of Intestinal Microflora in Colorectal Cancer Patients after Surgical Resection and Chemotherapy" was retracted in 2023. Reasons: signs of a paper mill; suspected computer-generated content; unreliable results or conclusions; concerns about the data.

### 2.8. Species Phenotype Analysis of Fecal Bacteria

By integrating the gene information of species in Integrated Microbial Genomes database (IMG, https://img.jgi.doe.gov/cgi-bin/m/main.cgi/m/main.cgi) [16], KEGG (https://www.kegg.jp/) [17], and PATRIC (https://www.patricbrc.org/) [18, 19] databases, the phenotypic characteristics of species were classified. According to the species annotation results of Greengene database (http://greengenes.secondgenome.com/) [20], the corresponding relationship of “species-gene-phenotype” was constructed, and the phenotype classification and abundance of samples were predicted by BugBase software (https://bugbase.cs.umn.edu/).

### 2.9. Functional Enrichment Analysis of Fecal Bacteria

IMG, PICRUSt2, SILVA, and other databases were used to construct the evolutionary tree. The reference species of OTU were selected according to the tree structure, and the “species-gene” relationship network was built by Functional Annotation of Prokaryotic Taxa (FAPROTAX, http://www.loucalab.com/archive/FAPROTAX) [21] and Tax4Fun (http://tax4fun.gobics.de/) [22] software. The count values of KO (Kyoto Encyclopedia of Genes and Genomes ontology) pathway in each sample were analyzed for direct comparison between groups.

### 2.10. Statistical Analysis

GraphPad Prism 7.0 software (San Diego, CA, USA) was used for data analysis. The Kruskal-Wallis (KW) rank sum test was used to analyze the difference of species richness among groups. Then, the Wilcoxon rank sum test and Welch's *t* test were used to test the difference between the two groups. *P* < 0.05 showed that there was significant difference between the groups.

## 3. Results

### 3.1. Clinical Situation of Colorectal Cancer Patients

The gastrointestinal tumors were identified by endoscopy and pathological staining (Figure 2). CRC patients included in the study collected intestinal flora samples before and after surgical eradication and after chemotherapy. The disease and treatment groups (12 samples) of 17 intestinal microbiological samples were collected from 5 cases of different CRC patients, including 3 men, 2 women, 3 colon cancer, and 2 rectal cancer. The clinical information of CRC patients is shown in Table 1.

### 3.2. Intestinal Bacterial Diversity in Patients with Colorectal Cancer before and after Treatment

A total of 1475040 original reads (an average of 86767.06 reads/sample) were obtained following quality control. The average effective data ratio was 80.93% (Table S1 and Figure S1). According to the statistics of total OTUs, the total number of intestinal bacteria in CRC patients increased significantly compared with the control group. There was no significant difference between CRC with CRC_O and CRC_C groups (Figure S2A). 402 of OTUs codistributed among the four groups (control, CRC, CRC_O, and CRC_C) were used for subsequent diversity studies (Figure S2B).

The article "Changes of Intestinal Microflora in Colorectal Cancer Patients after Surgical Resection and Chemotherapy" was retracted in 2023. Reasons: signs of a paper mill; suspected computer-generated content; unreliable results or conclusions; concerns about the data.

The results of alpha diversity analysis showed that the Chao1 index of CRC (*P* = 0.0079), CRC_O (*P* = 0.0159), CRC_C (*P* = 0.0357) had a higher level than that of the control group (Figure 3(a)), and the difference was statistically significant. There was no statistically significant change in Chao1 index among the CRC, CRC_O, and CRC_C groups (*P* > 0.05). The change trend of Observed_OTUs (Figure S3A) and ACE (Figure S3B) indexes was similar to that of Chao1 index. There was no significant difference in the Simpson (Figure 3(b)) and Shannon (Figure S3C) indexes between all study groups (*P* > 0.05) (Figure 3(c)).

Based on the distance of species evolution (Unweighted_unifrac index), UPGMA cluster tree and PCoA results showed that the sample distance was consistent with the grouping (Figures 4(a) and 4(b)). The ANOSIM test showed that there were significant differences among all groups (*P* = 0.001) (Figure S4A). Compared with the control group, the OTU composition based on Unweighted_unifrac distance of CRC (*P* = 0.008), CRC_O (*P* = 0.009), and CRC_C (*P* = 0.022) was significantly higher (Figure 4(c) and Figure S4A). Based on the Jaccard distance, beta diversity of gut flora in CRC_O and CRC_C was significantly lower than that of the control group (Figures 4(c)–4(e)). There was no significant difference in the CRC, CRC_O, and CRC_C groups (Figure 4(d)). The change of beta diversity based on Weighted_unifrac distance in each group was not statistically significant, and the change trend of beta diversity based on the Bray distance was similar to that of the Jaccard distance (Figure 4(d)). Then, the beta diversity of flora at different levels was analyzed. It was found that only the beta diversity based on the Jaccard distance at genus level was significantly reduced between the control and CRC_O groups (Figure S4C). These results indicated that the diversity of intestinal microflora in CRC patients increased significantly compared with the normal population, and surgery and chemical therapy failed to alleviate this trend. Surgical treatment had the potential to change the diversity of intestinal bacterial composition.

The article "Changes of Intestinal Microflora in Colorectal Cancer Patients after Surgical Resection and Chemotherapy" was retracted in 2023. Reasons: signs of a paper mill; suspected computer-generated content; unreliable results or conclusions; concerns about the data.

Notes are appended as follows:

Raw PE: Original pair-end reads logarithm,

Clean PE: High-quality pair-end reads logarithm after quality control filtration,

Raw Tags: Raw tags after overlap assembling,

Clean Tags: High-quality tags after tags filter,

Chimera: The number of chimeric tags detected in OTU clustering,

Effective Tags: The number of high-quality tags after removing the chimera, which is the effective tags for subsequent analysis,

Effective Ratio (%): Percentage of high-quality tags in original PE reads.

CON_1-CON_5 belongs to the control group; CC_1-CC_3 are samples from colon cancer patients, belonging to the CRC group; CCT0_1 and CCT0_2 are samples from colon cancer patient after operation treatment, belonging to the CRC_O group; CCT1_1 and CCT1_2 are samples from colon cancer patient after chemotherapy, belonging to the CRC_C group; RC_1 and RC_2 are samples from rectal cancer patients, belonging to the CRC group; RCT0_1 is sample from rectal cancer patient after operation treatment, belonging to the CRC_O group; RCT1_1 and RCT1_2 are samples from rectal cancer patient after chemotherapy, belonging to the CRC_C group.

### 3.3. Differences of Bacterial Phylogenetic Spectrum and Taxa in Colorectal Cancer Patients before and after Treatments

99%, 99.98%, 99.52%, 99.32%, and 92.47% of phylum, class, order, family, and genus were successfully annotated, but only 14.60% of species were annotated. *Firmicutes*, *Proteobacteria*, *Actinobacteria*, and *Bacteroides* constitute >90% of bacteria phyla in each group, showing basically consistent phylum relative abundance between groups (Figure 5(a)). The first three most abundant families in normal people were *Lachnospiraceae*, *Ruminococcaceae*, and *Enterobacteriaceae*. The most abundant family of CRC and CRC_O patients was *Enterobacteriaceae* and the second was *Veillonellaceae* (CRC) and *Bifidobacteriaceae* (CRC_O), followed by *Lachnospiraceae* (CRC) and *Ruminococcaceae* (CRC_O), respectively. *Lachnospiraceae* family is the most abundant in the CRC group, followed by *Enterobacteriaceae* family (Figure 5(b)). In genus level, the relative abundance of *Bifidobacterium* (13.87%) and *Escherichia_Shigella* (10.44%) in the control group was higher than other genera; the relative abundance of *Escherichia_Shigella* (31.53%) and *Megamonas* (14.15%) was higher in the CRC groups. In the CRC_C group, *Escherichia_Shigella* (15.86%) and *Ruminococcus*_gnavus (14.72%) were higher. The relative abundance of *Escherichia_Shigella* (39.49%) and *Bifidobacterium* (7.81%) was higher in the CRC_O group (Figure 5(c)).

The article "Changes of Intestinal Microflora in Colorectal Cancer Patients after Surgical Resection and Chemotherapy" was retracted in 2023. Reasons: signs of a paper mill; suspected computer-generated content; unreliable results or conclusions; concerns about the data.

LEFSE and IndVal were used to evaluate the differences of intestinal bacterial populations in CRC patients to determine significantly enriched bacterial taxa before and after treatment. Compared with the control group, the intestinal tract of CRC patients was enriched with *Negativicutes* class, *Clostridia* class, *Selenomonadales* order, *Clostridiales* order, *Veillonellaceae* family, and *Megamonas* genus (IndVal = 14.15) (*P* < 0.05, abundance > 10). And normal people was enriched with *Clostridia* class, *Negativicutes* class, *Clostridiales* order, *Selenomonadales* order, and *Blautia* genus (IndVal = 3.91) (*P* < 0.05, abundance > 2.5). Compared with the CRC group, the flora of CRC_C was enriched with *Verrucomicrobia* phylum, *Verrucomicrobiae* class, *Verrucomicrobiales* order, *Akkermansiaceae* family, and *Akkermansia* genus (*P* < 0.05, abundance > 9). The bacterial classification of the CRC_C group was similar to CRC. Compared with normal people, the microbiota of colorectal cancer patients showed different bacterial populations at the taxonomic level of phylum, class, order, family, genus, and species. Chemical therapy led to significant changes in intestinal bacterial populations of CRC patients at the levels of phylum, class, order, and family, but there was no significant difference in bacterial populations after radical surgery (Table 2 and Figure S5).

### 3.4. Effect of Surgery and Chemotherapy Treatment on Intestinal Microflora Phenotype in Patients with Colorectal Cancer

BugBase analyzed the bacterial phenotype of each group, and the results showed that the control group was mainly enriched in *Anaerobic* and *Gram_positive* phenotypes, while the CRC group was mainly enriched in *Anaerobic*, *Gram_positive*, and *Gram_negative* phenotypes. The CRC_C group was similar to the control group, and species were mainly enriched in *Anaerobic* and *Gram_positive* phenotypes. The CRC_O group was mainly enriched in the *Gram_negative* and contains mobile element phenotypes (Figure 6(a)). There was significant difference in *Aerobic* phenotype between groups (*P* = 0.031), but the difference only existed between the CRC and CRC_O groups. There was no significant difference in species phenotype between the CRC and control groups (Figure 6(b)). This indicated that the bacteria change of CRC_O group was related to *Aerobic* phenotype. The *Aerobic* germs in the CRC_O group were mainly distributed in the *Proteobacteria* phylum (Figure 6(c)). For the analysis of phenotypic function among groups, the increase of *Aerobic* phenotype led to the enhancement of respiration of sulfur compounds (Figure 6(d)).

### 3.5. Effect of Chemical Drugs and Surgical Treatment on Intestinal Flora Function in Patients with Colorectal Cancer

The change of bacterial composition affects its function in the intestine. Compared with normal people, intestinal bacteria in CRC patients significantly increased the biological pathway of lipopolysaccharide biosynthesis (*P* = 0.02915), phosphotransfer system (PTS) (*P* = 0.02222), D-arginine and D-ornithine metabolism (*P* = 0.03061), biotin metabolism (*P* = 0.01746), and so on (Figure 7(a)). After chemotherapy, the biological pathways of streptomycin biosynthesis (*P* = 0.02499) and polyketide sugar unit biosynthesis (*P* = 0.04511) of intestinal bacteria in CRC patients were significantly enhanced, and the ability of vitamin B6 metabolism (*P* = 0.02151) was weakened (Figure 7(b)). Compared with the intestinal bacterial function of CRC patients before treatment, the metabolism of xenobiology by cytochrome P450 (*P* = 0.00913) biological pathway was significantly enhanced after surgical eradication (Figure 7(c)).

The article "Changes of Intestinal Microflora in Colorectal Cancer Patients after Surgical Resection and Chemotherapy" was retracted in 2023. Reasons: signs of a paper mill; suspected computer-generated content; unreliable results or conclusions; concerns about the data.

### 3.6. Changes and Functions of Key Intestinal Bacteria in Colorectal Cancer Patients before and after Treatments

The marker intestinal bacteria of each group were identified based on the genus level. *Megamonas* (IndVal = 14.15) was the indicator and dominant genus of CRC patients, and its abundance was 103.49 times of that of the control group, while *Ruminocaceae_UCG-014* (IndVal = 3.85) was the dominant germ in the control group (Figure 8(a)). Both belong to *Firmicutes* phylum. The Pearson correlation between *Megamonas* and *Ruminocaceae_UCG-014* was weak (*P* > 0.05). *Prevotellaceae_UCG-001* genus in the CRC_O group was significantly higher (*P* = 0.045, fold = 97.58) than the CRC group (Figure 8(b)). Compared with CRC group, the most significant genera (*P* < 0.05) in the CRC_C group were Prevotellaceae_UCG-001 (IndVal = 0.062) and Tyzzerella_4 (IndVal = 0.027) of Pasteurellaceae family (Figure 8(c)).

There was positive correlation between *Megamonas* with *Megasphaera* (*r* = 0.625711, *P* = 0.007218) and *Ruminococcus_torques_group* (*r* = 0.533661, *P* = 0.027364) (Figure 9(a)). *Ruminocaceae_UCG-014* was mainly associated with *Lachnospiraceae nk4a136 group*, *Lachnospiraceae nd3007 group*, and *Ruminocacus_1* (*r* > 0.9, *P* < 0.001) (Figure 9(b)). They were mainly involved in metabolism, cellular processes, cancer, and other pathways. The KO pathway analysis showed that the intestinal microbial function of CRC patients was mainly involved in the biosynthesis and metabolism of glycans and the metabolism and degradation of terpenoids, polyketides, and heterobiotins. The biosynthesis of lipopolysaccharide, the biosynthesis of type II polyketide skeleton, and the degradation of nitrotoluene in CRC patients were significantly higher than those of normal people (fold > 2, *P* < 0.05) (Figure 9(c)). *Tyzzerella_4* was positively correlated with *Phascolarctobacterium* (*r* = 0.76, *P* = 0.00041), *Luminococcus gnavus group* (*r* = 0.74, *P* = 0.00065), and *Bacteroides* (*r* = 0.52, *P* = 0.031) in postoperative CRC patients (Figure 10(a)). These microfloras were mainly involved in adipocytokine signaling pathway, peroxisome, bile secretion, and fatty acid biosynthesis (fold > 1, *P* < 0.05) (Figure 10(b)). *Akkermansia* was positively correlated with six bacterial genus (*P* < 0.0001), including *Eubacterium ruminantium group* (*r* = 0.99), *Eubacterium nodatum group* (*r* = 0.97), and *Uba1819* (*r* = 0.85) in CRC patients after chemotherapy (Figure 10(c)). Analysis of these microbiota-related KO pathways in the CRC_C group showed that the rich genera mainly enhanced protein digestion and absorption in immune, digestive, and endocrine systems, renin-angiotensin system pathway, secondary bile acid biosynthesis, and adipocytokine signaling pathway (fold > 2, *P* < 0.05) (Figure 10(d)). After chemotherapy and surgical treatment, the adipocytokine signaling pathway, peroxisome, and bill secret KO pathway were significantly enhanced in CRC patients. Chemotherapy also significantly weakened the renin-angiotensin system, primary bile acid biosynthesis, nitrotoluene degradation, flagella assembly, etc. in the CRC group.

The article "Changes of Intestinal Microflora in Colorectal Cancer Patients after Surgical Resection and Chemotherapy" was retracted in 2023. Reasons: signs of a paper mill; suspected computer-generated content; unreliable results or conclusions; concerns about the data.

## 4. Discussion

There are more than 1000 kinds of bacteria in human intestinal tract, and the number is as high as 10 trillion. These bacteria form a barrier to protect the intestine and participate in the absorption and metabolism of nutrients. Bad dietary behavior affects the composition of intestinal flora, will disturb the normal metabolism of the body, and then affects the susceptibility of intestinal diseases, thus inducing inflammation, cancer, and other diseases. It is generally believed that the mechanism of action of intestinal flora on colorectal cancer is related to the increase of toxins produced by bacteria, the decrease of beneficial bacterial-derived metabolites, the destruction of epithelial barrier, the production of cancer-promoting compounds, and the change of intestinal flora or intestinal flora. Some studies have detected that species abundance is significantly downregulated in the intestine of CRC patients. However, in this study, the intestinal flora abundance and diversity of CRC patients are increased. In addition, there is no change in the composition of species structure. There seems to be a contradiction with the current research. This is proposed that the loss of specific beneficial bacteria or the serious loss of diversity among beneficial bacteria is the key to the occurrence of colorectal cancer.

The article "Changes of Intestinal Microflora in Colorectal Cancer Patients after Surgical Resection and Chemotherapy" was retracted in 2023. Reasons: signs of a paper mill; suspected computer-generated content; unreliable results or conclusions; concerns about the data.

In this study, the relative abundance differences of species composition in the colonies is further analyzed, and the significantly decreased abundance of *Ruminocaceae_UCG-014*, *Ruminococcus_1*, *Eubacterium_eligens*, and *Coprococcus_2* in colorectal cancer patients are found. Especially, *Rucocamace_UCG-014*, which belongs to the *Ruminocaceae* family, is related to fat metabolism. *Rucocamace_UCG-014* stimulates lactic acid metabolism to produce short-chain fatty acids and plays anti-inflammatory and anticancer roles. It is a kind of beneficial anaerobic bacteria [23–26]. The lack of *Ruminocaceae* leads to high intestinal inflammation and the high risk of cancer. The pathogenic bacteria *Allisonella* and *Megamonas* are significantly increased in CRC, which has the potential to trigger intestinal inflammation [27]. *Megamonas* belongs to *Clostridium* family in *Firmicutes* phylum [28], which is a kind of anaerobic bacteria. Especially *Megamonas* is positively correlated with lactic acid content and negatively correlated with acetate [29]. Some studies believe that *Megamonas* is the characteristic flora of lymph node metastasis of colorectal cancer and one of the main floras leading to abnormal metabolism of CRC. A medical research led by Han et al. [30] shows that *Megamonas* genus is a characteristic microorganism of the intestinal tract in colorectal cancer patients with lymph node metastasis, which is significantly associated with poor prognosis caused by lymph node metastasis. Through the analysis of KO functional pathway, it is found that the intestinal microflora of colorectal cancer is mainly related to lipopolysaccharide biosynthesis, biosynthesis of type II polysaccharide backbone, nitrotoluene degradation, etc. In addition, the function of renin-angiotensin system and primary bile acid biosynthesis is significantly reduced. *Megamonas* mediates the biosynthesis of lipopolysaccharide (LPS). High levels of lipopolysaccharide are detected in patients with irritable bowel syndrome and inflammatory bowel disease. The higher level of LPS is also increased of colorectal cancer incidence rate and the proliferation of tumor cells [31]. Therefore, the increased abundance of *Megamonas* leads to high level of LPS, which is a risk factor for cancer.

In addition, this study focused on the diversity and structural composition of intestinal flora in CRC patients before treatment, after surgical eradication, and after chemotherapy. This observation of intestinal colonies is useful for the identification of therapeutic effectiveness and recurrence. For example, the study of Jin et al. [9] detected that the intestinal microflora of 116 CRC patients before and after operation shows that there are significant differences between *Gemella*, *Tyzzerella 3*, *Unclassified Oxalobacteraceae*, *Howard Ella*, *Lawsonella*, and *Parascardovia*. In addition, high levels of *Fusobacterium nucleatum* (*F. nucleatum*) and *Bacteroides fragilis* (*B. fragilis*) significantly shortened the relapse-free survival. This is because these bacteria cause the decrease of butyrate metabolism, promote the proliferation of tumor cells, and ultimately increase the overall incidence rate and tumor survival rate [32]. *F. nucleatum* also activates autophagy to chemoresistance of colorectal cancer [33]. Therefore, intestinal flora of CRC patients after surgery and drug therapy improves lipid metabolism to a certain extent and thus participates in the prognosis of cancer patients.

The article "Changes of Intestinal Microflora in Colorectal Cancer Patients after Surgical Resection and Chemotherapy" was retracted in 2023. Reasons: signs of a paper mill; suspected computer-generated content; unreliable results or conclusions; concerns about the data.

The results in this study showed that there was no significant change in species diversity in the three stages (CRC, CRC_O, and CRC_C groups). There was no significant change in intestinal colony structure before and after surgical eradication, while chemotherapy affected the relative abundance of *Verrucomicrobia* phylum and subordinate microbiota. In fact, surgery and chemical drug treatment do not regulate the abundance of intestinal flora in CRC patients including *Megamonas* and *Ruminocaceae_UCG-014*. Relative abundance of *Prevotellaceae_UCG-001* in CRC patients is significantly increased after surgery, which is related to nutritional metabolism. *Prevotellaceae_UCG-001* promotes the metabolism of cholesterol and bile acids [34] and significantly reduces [35] in colitis animal models. Upregulation of *Prevotellaceae_UCG-001* promotes the production of short-chain fatty acids, improves intestinal microbial composition, regulates the immune regulatory activity related to intestinal flora, and maintains intestinal homeostasis [36]. *Akkermansia* genus is a kind of *Gram-negative* bacteria and a promising probiotic candidate [37, 38]. The results of a study in mice with colitis showed that the probiotics *Akkermansia* inhibits the occurrence of cancer [39]. *Akkermansia* is an effective colony marker for colon cancer treatment.

There are 5 CRC patients in this study, and the biological sample size is small, which needs to be further improved. In addition, the correlation between human genome and intestinal flora is ignored and does not fully explain the molecular mechanism of intestinal flora regulating colorectal cancer. This also needs to be improved in the future.

## 5. Conclusion

In this study, the abundance and diversity of intestinal flora in colorectal cancer patients are significantly higher than that of normal man. The abundance of *Prevotellaceae_UCG-001* is significantly decreased and *Megamonas* is significantly increased in CRC patients, which are involved in the biosynthesis of lipopolysaccharide and have a potential role in promoting colorectal cancer. However, chemical drug and surgical treatment do not alleviate the rise trend of intestinal flora abundance but reduce *Tyzzerella_4* and increase the proportion of *Akkermansia* to regulate intestinal immunity and metabolism.

The article "Changes of Intestinal Microflora in Colorectal Cancer Patients after Surgical Resection and Chemotherapy" was retracted in 2023. Reasons: signs of a paper mill; suspected computer-generated content; unreliable results or conclusions; concerns about the data.

## Figures and Tables

**Figure 1:** Collection, storage, and handle of intestinal microbiological samples. The process is the overall step of 16S sequencing, including aseptic collection of fecal samples, centrifugal enrichment of bacteria, DNA extraction, construction of DNA library, and DNA sequencing.

**Figure 2:** Endoscopic examination of colorectal cancer tissue. The lesion site of the colon (a) and rectum (c) under endoscope. Hematoxylin and eosin (H&E) staining results of colon (b) and rectal (d) cancer tissues under light microscope (100x).

**Figure 3:** Alpha diversity of intestinal flora before and after treatment of colorectal cancer. (a–b) Chao1 and Simpson index results and (c) heat map of the Wilcoxon test analysis results of alpha diversity indexes.

**Figure 4:** Beta diversity analysis of intestinal bacteria before and after treatment of colorectal cancer. Unweighted pair group method with arithmetic mean (UPGMA) cluster tree (a) and principle coordinate analysis (PCoA) plot based on Unweighted_unifrac distances show distinct bacterial community clusters between the control and CRC patients before and after treatments (b), PCoA plot shows distinct bacterial community clusters based on Jaccard (c), the heat map shows the ANOSIM test results of beta diversity indexes (Unweighted_unifrac, Weighted_unifrac, Bray, and Jaccard) among each group (d), and box diagram shows the OTU diversity based on the Jaccard distance of each group (e).

**Figure 5:** Stacking map of species distribution at phylum (a), family (b), and genus (c) levels of each group.

**Figure 6:** Intestinal bacteria phenotype and function analysis of colorectal cancer patients before and after treatment. (a) The phenotypic distribution of each group, (b) the analysis of phenotypic differences among groups, (c) the distribution of aerobic species, and (d) the analysis of KO pathway.

**Figure 7:** The difference of intestinal bacterial function in patients with colorectal cancer before and after treatment. Panel (a) shows the KO pathway difference of intestinal bacteria between healthy people and colorectal cancer patients, with the Welch *t* test *P* less than 0.05, while panels (b) and (c) show the difference after chemotherapy and operation, respectively.

The article "Changes of Intestinal Microflora in Colorectal Cancer Patients after Surgical Resection and Chemotherapy" was retracted in 2023. Reasons: signs of a paper mill; suspected computer-generated content; unreliable results or conclusions; concerns about the data.

**Figure 8:** Genera with indicative significance in the intestine of colorectal cancer patients before and after treatments. Panel (a) shows the genera that are significantly abundant between the CON and CRC groups tested by the Wilcoxon rank method (*P* < 0.05), while panels (b) and (c) show the genera between the CRC_O group and CRC_C group with the CRC group, respectively.

**Figure 9:** The predominant intestinal flora interaction of healthy people (a) and colorectal cancer patients (b) and functional difference analysis (c).

**Figure 10:** The predominant intestinal flora interactions (a, c) and their functional differences (b, d) in colorectal cancer patients after surgery and chemical drug therapy.

**Table 1:** Statistics of clinical data of colorectal cancer patients.

Patients	Mean ± SD
Age (year)	58.20 ± 12.09
Gender (*n* = 5)	
Female	2
Male	3
Colorectal cancer	
Colon cancer	3
Rectal cancer	2
Tumor size (cm^3^)	28.23 ± 20.91
Clinical stage	
I	1
II	1
III	2
IV	1
MMR (*n* = 5)	1
Ki-67 (+)	62.00 ± 16.00%
Chemotherapy methods	
	Tegafur+irinotecan
	Tegafur+calcium folinate+oxaliplatin
	Tegafur+irinotecan+calcium folinate+oxaliplatin
Times of chemotherapy	4.80 ± 1.64
Lymphatic metastasis	3

MMR indicates CRC patients with Lynch syndrome who carry a mismatch repair (MMR) gene mutation.

**Table 2:** The results of bacterial classification differences in each group based on LEFSE method (*P* < 0.05).

Levels	Control	CRC	CRC_C	CRC_O
Phylum	—	Verrucomicrobia, Synergistetes	Verrucomicrobia	—
Class	—	Acidimicrobiia, Deltaproteobacteria, Synergistia, and Verrucomicrobiae	Verrucomicrobiae	—
Order	Phycisphaerales, Gemmatales, and Desulfuromonadales	Propionibacteriales, Desulfovibrionales, Corynebacteriales, Synechococcales, Synergistales, IMCC26256, and Verrucomicrobiales	Chloroplast, Verrucomicrobiales	—
Family	Rhizobiaceae, Bacillaceae, Candidatus_Melainabacteria_bacterium_MELA1, Coriobacteriales_Incertae_Sedis, Gemmataceae, Geobacteraceae, and Phycisphaeraceae	Akkermansiaceae, Aerococcaceae, Synergistaceae, Cyanobiaceae, and Desulfovibrionaceae	Akkermansiaceae, Clostridiaceae_1	—
Genus	Bacillus, Coprococcus_2, Coprococcus_1, Ruminococcus_1, Lachnospira, Eubacterium_hallii_group, Fusicatenibacter, Lachnospiraceae_UCG_003, Adlercreutzia, Erysipelotrichaceae_UCG_003, GCA_900066575, Prevotella_2, SM1A02, Ruminococcaceae_UCG_014, Eubacterium_ventriosum_group, Mitsuokella, Geobacter, Senegalimassilia, Lachnospiraceae_UCG_010, Ruminococcaceae_UCG_003, Ruminococcaceae_UCG_002, Faecalibacterium, Lachnospiraceae_ND3007_group, Lachnospiraceae_NK4A136_group, Fimbriiglobus, Lachnospiraceae_UCG_001, and Phyllobacterium	Erysipelatoclostridium, Abiotrophia, Curvibacter, Ralstonia, Bilophila, Akkermansia, and Burkholderia_Caballeronia_Paraburkholderia	Eubacterium_ruminantium_group, Akkermansia	—
Species	Clostridium_perfringens_CPE_str_F4969, Bifidobacterium_animalis, Veillonella_magna, Ruminococcus_bicirculans, Alistipes_inops, Coprococcus_sp_DJF_B005, and Lachnospiraceae_bacterium_TF01_11	GCA_900066225, Pyramidobacter, Hungatella, Eubacterium_sp_Marseille_P3202, Bacteroides_vulgatus, Parabacteroides_distasonis, Hungatella_hathewayi, Clostridium_symbiosum_ATCC_14940, Erysipelatoclostridium_ramosum, Akkermansia_muciniphila, Emergencia_timonensis, and Corynebacterium_afermentans_subsp_afermentans	—	—

The article "Changes of Intestinal Microflora in Colorectal Cancer Patients after Surgical Resection and Chemotherapy" was retracted in 2023. Reasons: signs of a paper mill; suspected computer-generated content; unreliable results or conclusions; concerns about the data.

## Data Availability

The data used to support the findings of this study are available from the corresponding author upon request.

## Abbreviations

CRC: Colorectal cancer
KEGG: Kyoto Encyclopedia of Genes and Genomes
KO: Kyoto Encyclopedia of Genes and Genomes Ontology
OTU: Operational tax unit
UPGMA: Unweighted pair group method with arithmetic mean
PCoA: Principal coordinate analysis
NMDS: Nonmetric multidimensional scaling
IndVal: Indicator values
IMG: Integrated Microbial Genomes
FAPROTAX: Functional Annotation of Prokaryotic Taxa
KW: Kruskal-Wallis rank sum test
CON: Control
CC: Colon cancer
CCT: Colon cancer patients after treatment
RC: Rectal cancer
RCT: Rectal cancer patients after treatment.

## Supplementary Materials

Supplementary 1 Table S1: pretreatment and quality control of sequencing data.

Supplementary 2 Figure S1: effective reading percentage (A) and number (B) of 16S sequencing of microorganisms in each sample. Reads QC filter, low quality reads; nonoverlap, reads that cannot be spliced into tags; tag QC filter, tags that do not pass “tag filtering”; and effective tags, effective tags for subsequent analysis.

Supplementary 3 Figure S2: histogram of changes in total OTUs (A) and Venn diagram of total OTU distribution (B) of intestinal flora in patients with colorectal cancer before and after treatments. ^∗∗^ indicates *P* < 0.01 via comparing with the control group.

Supplementary 4 Figure S3: alpha diversity analysis dilution curve. (A-C) Observed_OTUs, ACE, and Shannon indexes. OTUs: operational tax units. ACE, Abundance-based Coverage Estimator, indicates bacterial abundance.

Supplementary 5 Figure S4: box diagram of the ANOSIM test results of flora beta diversity based on the unweighted distance (A) and Jaccard distance (B) in CRC patients before and after treatments. And the heat map (C) shows the ANOSIM test results of flora beta diversity based on the Jaccard distance at different levels (phylum, class, order, family, genus, and species).

The article "Changes of Intestinal Microflora in Colorectal Cancer Patients after Surgical Resection and Chemotherapy" was retracted in 2023. Reasons: signs of a paper mill; suspected computer-generated content; unreliable results or conclusions; concerns about the data.

Supplementary 6 Figure S5: the distribution of bacterial clusters in CRC patients before and after treatment. The bar chart shows the bacterial structure composition at the (A) phylum, (B) order, (C) class, (D) family, and (D) genus levels with significant differences among the groups tested by Kruskal-Wallis (KW) method (*P* < 0.05).
